# MicroRNA-488 inhibits tongue squamous carcinoma cell invasion and EMT by directly targeting ATF3

This article has been retracted.

**DOI:** 10.1186/s11658-018-0094-0

**Published:** 2018-06-18

**Authors:** Bingxia Shi, Wei Yan, Guolin Liu, Yanjun Guo

**Affiliations:** Oral and Maxillofacial Surgery, Cangzhou Central Hospital, No. 16 Xinhua West Road, Cangzhou, Hebei 061000 People’s Republic of China

**Keywords:** Tongue squamous carcinoma, MicroRNA-488, Activating transcription factor 3, Invasion, Epithelial–mesenchymal transition

## Abstract

**Background:**

It has been reported that the expression of activating transcription factor 3 (ATF3) is closely associated with both microRNA (miRNA) processing and the progress of many cancers. Our study aimed to explore the interaction between ATF3 and miR-488 in tongue squamous cell carcinoma (TSCC).

**Methods:**

Quantitative real-time PCR was performed to detect the levels of ATF3 and miR-488 in TSCC tissues and cell lines. Cell invasion and epithelial–mesenchymal transition (EMT) were assessed to determine the biological functions of miR-488 and ATF3 in TSCC cells. The mRNA and protein levels of ATF3 were measured using quantitative RT-PCR and western blotting. Luciferase assays were performed to validate ATF3 as an miR-488 target in TSCC cells.

**Results:**

We found that the level of miR-488 significantly decreased and the expression of ATF3 significantly increased in TSCC tissues and cell lines. A low level of miR-488 was closely associated with increased expression of ATF3 in TSCC tissues. Introducing miR-488 significantly inhibited the invasion and EMT of TSCC cells, and knockdown of miR-488 promoted both processes. The bioinformatics analysis predicted that ATF3 is a potential target gene of miR-488. The luciferase reporter assay showed that miR-488 could directly target ATF3. ATF3 silencing had similar effects to miR-488 overexpression on TSCC cells. Overexpression of ATF3 in TSCC cells partially reversed the inhibitory effects of the miR-488 mimic.

**Conclusion:**

miR-488 inhibited cell invasion and EMT of TSCC cells by directly downregulating ATF3 expression.

## Background

Tongue squamous cell carcinoma (TSCC) is one of the most common malignancies of the mouth, accounting for over 90% of mouth tumors. It poses a serious threat to human life and health [1, 2]. Despite many advances in treatment, including radical surgery, radiotherapy and neo-adjuvant chemotherapy, TSCC is still associated with a poor prognosis. Because of its strong local invasion and high rate of lymph node metastasis, the five-year survival rate of patients is only ~ 50% [3–5]. It is therefore critical to investigate the mechanism of invasion and finding a more effective strategy to therapy TSCC.

Activating transcription factor 3 (ATF3), a member of the mammalian activation transcription factor family of transcription factors, also called the cAMP responsive element-binding (CREB) protein family [6], has been linked with the biological behaviors of multiple cancers, including breast cancer [7], diffuse large B-cell lymphoma [8], prostate cancer [9, 10], esophageal squamous cell carcinoma [11, 12], and Hodgkin lymphoma [13]. However, the exact role of ATF3 remains controversial in cancer development and progression, since this adaptive-response gene has been identified as both an oncogene and a tumor-suppressor gene [14].

The role of ATF3 in TSCC is still unknown. This present study was designed to examine the effect of ATF3 overexpression on the biological behaviors of TSCC cells, to provide new insights into the role of ATF3 in TSCC.

MicroRNAs (miRNAs) are small non-coding RNAs that regulate the translation of many genes by binding to the untranslated region (3’UTR) of target mRNAs. They are involved in a variety of physiological and pathological processes, including cancer development [15, 16]. Accumulating evidence shows that miRNAs are aberrantly expressed in many types of cancer, including TSCC, with some functioning as tumor-suppressor genes and others as oncogenes [17, 18].

Distinct miRNAs are reportedly directly involved in carcinogenesis and progression of TSCC through the regulation of cell proliferation, apoptosis, invasion and drug sensitivity [19–21]. For example, Sun et al. showed that miR-137 suppresses the proliferation, migration and invasion of TSCC [19]. Hou et al. showed that miR-509 acts as a tumor suppressor in TSCC by targeting epidermal growth factor receptor [20]. Wu et al. suggested that miR-802 plays a tumor suppressive role in TSCC by directly targeting MAP2K4 [21]. However, the expression and role of miR-488 in TSCC remains unclear.

We found that the expression of ATF3 is markedly upregulated in TSCC tissues and cell lines. However, its effects in TSCC remain unclear. Using the online database microRNA.org, we found that miR-488 might directly target ATF3, and that it was considered a tumor suppressor in many cancers, including non-small-cell lung cancer and hepatocellular carcinoma [22, 23]. We also confirmed significant downregulation of miR-488 in TSCC tissues and cells. Overexpression of miR-488 inhibited invasion and epithelial–mesenchymal transition (EMT) of TSCC cells. Moreover, we found that ATF3 was the direct target of miR-488 in TSCC. Restoration of ATF3 reversed the inhibitory effects of miR-488. Therefore, our results showed critical roles for miR-488 in the pathogenesis of TSCC and suggested its possible application in tumor treatment.

## Methods

### Human tissue samples

Human TSCC tissues (*n* = 20) and their adjacent non-cancer tissues (*n* = 10) were collected from patients at the Cangzhou Central Hospital between May 2015 and May 2017. All samples were immediately frozen in liquid nitrogen for subsequent quantitative RT-PCR analysis. All study procedures were approved by the Research Ethics Committee of the Cangzhou Central Hospital. Informed consent was given by all participants.

### Cell culture

Human tongue cancer cell lines UM1, TCA8113, Cal27, SCC1 and SCC25 were obtained from the American Type Culture Collection (ATCC). The cells were cultured in Dulbecco’s modified Eagle’s medium (DMEM; GIBCO) supplemented with 10% fetal bovine serum (FBS; GIBCO). Human normal oral keratnocyte cell culture (NHOK) was purchased from ATCC and cultured in DMEM/F12 medium supplemented with 10% FBS. All cell lines were maintained at 37 °C in 5% CO_2_.

### Transient transfection

The miR-488 mimics, miR-488 inhibitors, negative control (NC), siRNA for ATF3 (si-ATF3) and siRNA-negative control (si-NC) were synthesized and purified by Gene-Pharma. The ATF3-overexpression plasmid was generated by inserting ATF3 cDNA into a pcDNA3.1 vector. This plasmid was sequenced and confirmed by Gene-Pharma. miR-488 mimics, miR-488 inhibitors, si-ATF3 and ATF3-overexpression plasmid were transfected using Lipofectamine 3000 reagent (Invitrogen) per the manufacturer’s protocols. Cells (10^7^/well) were transfected for 48 h in the 6 well-plate, and total RNA and protein were collected.

### RNA extraction and quantitative real-time PCR

Total RNA was extracted from tissues and cells using Trizol reagent (Invitrogen) per the manufacturer’s protocol. Reverse transcription was performed using miScript Reverse Transcription Kit (QIAGEN) and the QuantiTect SYBR Green RT-PCR Kit (QIAGEN) was used for quantitative real-time PCR analysis with the ABI 7500 Fast Real-Time PCR System (Applied Biosystems) following the manufacturer’s instructions. The relative expression levels of miR-488, ATF3, N-cadherin, E-cadherin and vimentin were normalized to those of internal control U6 or GAPDH using the comparative delta CT (2^-ΔΔCt^) method. Each sample was analyzed in triplicate and the mean expression level was calculated. Prime sequences are shown in Table 1.

**Table 1:** Sequence of primers for quantitative RT-PCR

Gene	Primer sequence
ATF3	F: 5’-CCTCTGCGCTGGAATCAGTC-3′
	R: 5’-TTCTTTCTCGTCGCCTCTTTTT-3′
E-cadherin	F: 5’-TACACTGCCCAGGAGCCAGA-3′
	R: 5’-TGGCACCAGTGTCCGGATTA-3′
N-cadherin	F: 5′- TCAGGCGTCTGTAGAGGCTT-3’
	R: 5′- ATGCACATCCTTCGATAAGACTG-3’
Vimentin	F: 5’-GACGCCATCAACACCGAGTT-3’
	R: 5’-CTTTGTCGTTGGTTAGCTGGT-3’
U6	F: 5’-CTCGCTTCGGCAGCACA-3’
	R: 5’-AACGCTTCACGAATTTGCGT-3’
GAPDH	F: 5’-GAGTCAACGGATTTGGTCGTATTG-3’
	R: 5’-CCTGGAAGATGGTGATGGGATT-3’

### In vitro invasion assay

The transwell invasion assay was carried out by adding 100 μl Matrigel (BD Bioscience) into the upper chamber of a 24-well transwell plate and placing cells (10^6^/well) onto the Matrigel for 24 h. The non-invasive cells that were above the faces of the membranes were then removed and the invasive cells were fixed with methanol for 15 min, and then stained with 0.1% crystal violet for 20 min. Cells were imaged at least five grids per field. The membranes were then rinsed with 30% glacial acetic acid. Finally, the washing solution was examined at 540 nm to count the number of TCA8113 cells. All assays were independently repeated three times.

### Protein extraction and western blot analysis

Transfected cells were solubilized with RIPA lysis buffer (Beyotime Biotechnology) containing protease inhibitors (Millipore). Protein concentration was measured using a BCA protein assay kit (Beyotime Biotechnology). Equal amounts of protein were separated with 12% SDS-PAGE and transferred to polyvinylidene difluoride (PVDF) membranes (Millipore). The membranes were then blocked with 5% non-fat milk in TBST for 1 h at room temperature, followed by incubation with primary antibodies of ATF3, MMP-2, MMP-7, MMP-9, TIMP-1, TIMP-2 (Abcam), E-cadherin, N-cadherin and vimentin (Cell Signaling Technology Inc.) overnight at 4 °C. Subsequently, the membranes were washed with TBST three times and probed with the corresponding horseradish peroxidase-conjugated secondary antibodies (Cell Signaling Technology Inc.) for 2 h at room temperature. ECL reagent (Pierce) was used to detect the signals on the membranes.

### Luciferase reporter assay

The luciferase reporter vectors (pGL3-ATF3–3’UTR WT and pGL3-ATF3–3’UTR MUT) were synthesized by GenePharma. TCA8113 cells were seeded into 24-well plates and transfected with pGL3-ATF3–3’UTR WT or pGL3-ATF3–3’UTR MUT, along with miR-488 mimics or NC using Lipofectamine 2000 per the manufacturer’s instructions. After transfection for 48 h, luciferase reporter assays were performed with the Promega Dual-Luciferase Reporter Assay System. The relative firefly luciferase activities were measured by normalizing to renilla luciferase activities.

### Statistical analysis

The data were expressed as the means ± standard error of the mean (S.E.M.). The number of independent experiments was represented by “n”. The relationship between miR-488 and the clinicopathological characteristics was tested using the chi-square test. Correlations between miR-488 and ATF3 mRNA levels were analyzed using Pearson’s correlation coefficient. Multiple comparisons were performed using one-way ANOVA followed by Tukey’s multiple-comparison test. Two-tailed Student’s *t*-test was used for other comparisons. *p* < 0.05 was considered statistically significant.

## Results

### High expression of ATF3 correlates with low levels of miR-488 in TSCC tissues and cells

We used quantitative RT-PCR to detect the levels of ATF3 in TSCC tissues and cell lines. The results showed that the mRNA level of ATF3 was significantly higher in TSCC tissues than in the adjacent tissues (Fig. 1a). We also determined the mRNA level of ATF3 in five TSCC cell lines (UM1, TCA8113, Cal27, SCC1 and SCC25) and a human normal oral keratnocyte cell culture (NHOK). The level of ATF3 in TCA8113 cells was higher than that in the other four TSCC cell lines or in NHOK (Fig. 1b).

**Fig. 1:** The expressions of ATF3 and miR-488 in TSCC tissues and cell lines. **a** Quantitative RT-PCR analysis of ATF3 expression in TSCC tissues (*n* = 30) and adjacent normal tissues (*n* = 10). Transcript levels were normalized to GAPDH expression. **b** Relative ATF3 expression analyzed via quantitative RT-PCR in five TSCC cell lines normalized to GAPDH (*n* = 6). **c** Quantitative RT-PCR analysis of miR-488 level in TSCC tissues and adjacent normal tissues. Transcript levels were normalized to U6 level. **d** Relative miR-488 level analyzed via quantitative RT-PCR in five TSCC cell lines normalized to U6 (n = 6). **e** Pearson’s correlation analysis of the relative expression levels of miR-488 and the relative ATF3 mRNA levels in TSCC tissues. All data are presented as means ± SEM. *p < 0.05, **p < 0.01, ***p < 0.001 vs. normal tissues or NHOK

Using the online database microRNA.org, we found that miR-488 may directly target ATF3. Our findings demonstrated that the level of miR-488 in the TSCC tissues was significantly lower than in the adjacent tissues (Fig. 1c). We also confirmed that miR-488 expression was lower in TCA8113 cells than that in the other four TSCC cell lines (Fig. 1d). Therefore, TCA8113 cells were used in the following experiments.

To determine whether the expression of ATF3 was associated with miR-488 in TSCC, Pearson’s correlation analysis was performed. It revealed a significant inverse correlation between ATF3 and miR-488 in TSCC tissues (Fig. 1e). From the above data, we predicted that ATF3 might be negatively regulated by miR-488.

### Knockdown of ATF3 inhibited invasion and EMT of TSCC cells

To study the effects of ATF3 on TSCC cells, the cell proliferation, invasion and EMT were estimated in TCA8113 cells after transfection with si-NC or si-ATF3 for 48 h. The quantitative RT-PCR and western blot analyses showed that the ATF3 expression significantly decreased in TCA8113 cells transfected with si-ATF3 for 48 h compared to the si-NC group (Fig. 2a). Transwell assays suggested that decreased ATF3 expression inhibited the invasive ability of TCA8113 cells (Fig. 2b). Moreover, western blot and ELISA assays demonstrated that silencing ATF3 dramatically downregulated the expressions of MMP-2, MMP-7 and MMP-9 (Fig. 2c), and upregulated TIMP-1 and TIMP-2 expressions (Fig. 2c). Knockdown of ATF3 significantly increased the expression of the epithelial marker E-cadherin and decreased the expressions of the mesenchymal markers N-cadherin and vimentin at both the mRNA and protein levels in TCA8113 cells (Fig. 3a), contributing to inhibition of EMT (Fig. 2d).

**Fig. 2:** The effects of ATF3 silencing on invasion and EMT in TSCC cells. TCA8113 cells were transfected with si-ATF3 or si-NC. **a** The mRNA and protein expressions of ATF3 were determined via quantitative RT-PCR and western blot, respectively. **b** Invasion was assessed via transwell assay. **c** The protein expressions of MMP-2, MMP-7 MMP-9, TIMP-1 and TIMP-2 were assessed via western blot and ELISA assays. **d** The expressions of E-cadherin, N-cadherin and vimentin were determined via quantitative RT-PCR and western blot assays, respectively. All data are presented as means ± SEM, *n* = 6. ^#^*p* < 0.05, ^##^*p* < 0.01 vs. si-NC

**Fig. 3:** ATF3 is a direct target of miR-488. TCA8113 cells were transfected with miR-488 mimic or inhibitor for 48 h. **a** Schematic representation of ATF3 3’UTRs showing putative miRNA target site. **b** The analysis of the relative luciferase activities of ATF3-WT and ATF3-MUT. **c** The mRNA and protein expressions of ATF3 were determined via quantitative RT-PCR and western blot, respectively. All data are presented as means ± SEM, *n* = 6. ^##^*p* < 0.01, ^###^*p* < 0.001 vs. miR-NC

### miR-488 directly targeted ATF3 3’UTR

Using microRNA.org, we identified an miR-488 binding site in the 3’UTR of ATF3 (Fig. 3a). To validate whether ATF3 is a direct target of miR-488, luciferase plasmids containing the potential ATF3 miR-488-binding sites (WT) or a mutated ATF3 3’UTR were constructed (Fig. 3a). Overexpression of miR-488 inhibited WT ATF3 reporter activity but not the activity of the mutated reporter construct in TCA8113 cells, demonstrating that miR-488 could specifically target the ATF3 3’UTR by binding to the seed sequence (Fig. 3b). Next, we confirmed the results at the mRNA and protein levels. Introduction of miR-488 could significantly decrease the expression of ATF3, whereas knockdown of miR-488 increased the ATF3 expression in TCA8113 cells (Fig. 3c). These data indicate that miR-488 directly regulated ATF3 expression in TSCC cells through 3’UTR sequence binding.

### The effects of miR-488 on invasion of TSCC cells

After transfection with a miR-488 mimic or an inhibitor, the quantitative RT-PCR analysis showed that the expression of miR-488 was respectively significantly upregulated or downregulated (Fig. 4a). These data demonstrated that we efficiently enhanced and reduced miR-488 expression, respectively, in TCA8113 cells.

**Fig. 4:** The effects of miR-488 on invasion and related molecules in TSCC cells. TCA8113 cells were transfected with miR-488 mimic or inhibitor for 48 h. **a** Invasion was assessed using a transwell assay. **b** The protein expressions of MMP-2, MMP-7, MMP-9, TIMP-1 and TIMP-2 were determined using western blot and ELISA assays. All data are presented as means ± SEM, *n* = 6. ^#^*p* < 0.05, ^##^*p* < 0.01, ^###^*p* < 0.001 vs. miR-NC

To study the role of miR-488 in the invasion of TSCC cells, we evaluated the invasive capacities of TCA8113 cells transfected with a miR-488 mimic or an inhibitor using transwell invasion assays. The transwell assays illustrated that the invasion of TCA8113 cells was remarkably suppressed in the miR-488 mimic group compared to the NC group, but was significantly promoted in the miR-488 inhibitor group compared to the NC group (Fig. 4b). These findings showed that miR-488 might play a critical role in the inhibition of TSCC cell invasion.

The balance between MMPs and TIMPs is known to play an important role of invasion by stimulating the degradation of the ECM in cancer cells and is associated with enhanced tumor metastatic potential. Our ELISA and western blot assays indicated that the total secretion of MMP-2, MMP-7 and MMP-9 in the culture supernatants and the expressions of MMP-2, MMP-7 and MMP-9 were evidently decreased by the overexpression of miR-488 in TCA8113 cells. The total secretion of TMIP-1 and TIMP-2 and the protein expressions of TMIP-1 and TIMP-2 significantly increased (Fig. 4c and d). However, the knockdown of miR-488 could enhance the secretion and protein expressions of MMP-2, MMP-7 and MMP-9 and reduce the secretion and protein expressions of TMIP-1 and TMIP-2 (Fig. 4c and d).

Our findings suggest that the downregulation of MMP-2, MMP-7 and MMP-9 and the upregulation of TMIP-1 and TMIP-2 might be the mechanisms contributing to the inhibitory effect of the miR-488 mimic on the invasion of TCA8113 cells.

### The effects of miR-488 on EMT in TSCC cells

For further study, we examined the effect of miR-488 on the expressions of EMT markers at the protein and mRNA levels in TSCC cells. Overexpression of miR-488 could dramatically enhance the expression of E-cadherin and reduce the expressions of N-cadherin and vimentin in TCA8113 cells (Fig. 5). However, the miR-488 inhibitor had the opposite effects on the expressions of these EMT markers (Fig. 5). Our data suggest that miR-488 upregulation significantly inhibited the invasion and EMT of TSCC cells. These findings reveal that the overexpression of miR-488 could inhibit the EMT of TSCC cells. Consequently, miR-488 overexpression had similar effects to ATF3 silencing in TSCC cells.

**Fig. 5:** The effects of miR-488 on the expressions of EMT-related molecules in TSCC cells. TCA8113 cells were transfected with miR-488 mimic or inhibitor for 48 h. The mRNA and protein expressions of E-cadherin, N-cadherin and vimentin were determined via quantitative RT-PCR and western blot, respectively. All data are presented as means ± SEM, *n* = 6. ^#^*p* < 0.05, ^##^*p* < 0.01, ^###^*p* < 0.001 vs. miR-NC

### Overexpression of ATF3 markedly reversed the effects of miR-488 upregulation on the invasion and EMT of TSCC cells

To determine whether miR-488 targeting ATF3 was responsible for inhibiting the invasion and EMT of TSCC cells, we constructed an expression vector that encoded the entire ATF3 coding sequence but lacked the 3’UTR. Then, we co-transfected this vector (pcDNA-ATF3) or its negative control (pcDNA3.1) with miR-488 mimic or NC into TCA8113 cells (Fig. 6a). We found that enhanced ATF3 expression partially reversed the inhibitory effect of miR-488 upregulation on the invasion of TSCC cells (Fig. 6b). Overexpression of ATF3 significantly upregulated the expressions of MMP-2, MMP-7 and MMP-9 (Fig. 6c) and downregulated TIMP-1 and TIMP-2 expressions compared with the miR-488 mimic group (Fig. 6c). Moreover, increased ATF3 expression promoted the EMT of TCA8113 cells transfected with miR-488 mimic (Fig. 6d). Therefore, the inhibitory effects of miR-488 were partially reversed by ATF3 overexpression.

**Fig. 6:** Overexpression of ATF3 partially promoted cell proliferation, invasion and EMT in miR-488-overexpressing TSCC cells. TCA8113 cells were transfected with either miR-488 mimic with or without pcDNA-ATF3 vector. **a** The mRNA and protein expressions of ATF3 were determined via quantitative RT-PCR and western blot assays, respectively. **b** Invasion was assessed using a transwell assay. **c** The protein expressions of MMP-2, MMP-7 MMP-9, TIMP-1 and TIMP-2 were assessed using ELISA assays. **d** The expressions of E-cadherin, N-cadherin and vimentin were determined via quantitative RT-PCR and western blot assays. All data are presented as means ± SEM, *n* = 6. ^#^*p* < 0.05, ^##^*p* < 0.01, ^###^*p* < 0.001 vs. pcDNA3.1 + miR-448 mimic

These results clearly confirmed that miR-488 inhibited cell invasion and EMT of TSCC cells and that this occurred due to miR-488 targeting and downregulating ATF3.

## Discussion

In molecular biology, ATF is a group of bZIP transcription factors that act as homodimers or heterodimers with a range of other bZIP factors [24]. Currently, seven members have been identified in the ATF family: ATF1, ATF2, ATF3, ATF4, ATF5, ATF6 and ATF7 [24]. ATF1 has been linked to multiple cancers, such as clear cell sarcoma [25], melanoma [26] and angiomatoid fibrous histiocytoma [27]. ATF2 has been found to play a dual role in tumorigenesis [28]. ATF4, which is more highly expressed in cancers than in normal tissues and regulates processes relevant to cancer progression, has been identified as a potential therapeutic target in cancers [29]. ATF5, a transcription factor closely related to cell apoptosis, differentiation and development, may be a promising biomarker for rectal cancer [30] and neural tumors [31] and a therapeutic target for pancreatic cancer [32]. ATF5 was also reported to enhance radioresistance and malignancy in cancer cells [33]. ATF6, a constitutively expressed, endoplasmic reticulum (ER) membrane-anchored transcription factor, is associated with liver cancer [34], breast cancer [35], prostate cancer [36], colonic neoplasm [37] and soft tissue sarcoma [38]. ATF7, a novel bZIP protein that interacts with PTP4A1 [39], was recently identified as a favorable factor for survival of patients with colorectal cancer [40].

ATF3 was found to act as an oncogene as well as a tumor suppressor [39]. Many studies support an oncogenic role of ATF3 in breast cancer, prostate cancer, Hodgkin lymphoma and colon cancer. However, there is also much evidence proving that AFT3 inhibits the development of prostate cancer, colorectal cancer and ovarian cancer [41]. A previous study reported that activation of the SAPK/JNK stress pathway could upregulate its downstream effector ATF3 [42].

Here, the expression of ATF3 were significantly upregulated in TSCC tissues compared to non-cancerous tissues. Up to now, several independent studies have reported that ATF3 expression is closely associated with many kinds of cancers. However, the effects of ATF3 on TSCC are still poorly understood. In this study, the expression of ATF3 was significantly increased in TSCC tissues and cell lines. Moreover, inhibition of ATF3 could dramatically suppress the invasion of TSCC cells.

Next, related genes such as MMPs and TIMPs were also assessed. Previous reports have showed that others transcription factors and other types of mediators, such as H19, FoxM1 and MAGE-A10, have also demonstrated effects on EMT in TSCC [43–45]. Here, our data indicated that knockdown of ATF3 could significantly inhibit invasion and EMT of TSCC cells by decreasing the expressions of MMP-2, MMP-7, MMP-9, N-cadherin and vimentin, and increasing the expressions of TIMP-1, TIMP-2 and E-cadherin.

miRNAs play crucial roles in the regulation of diverse target mRNAs at the level of mRNA degradation or translation. Increasingly, evidence suggests that miRNAs are involved in multiple biological processes and have an essential role in the regulation of genes during cancer development, progression and metastasis [46, 47]. It has been reported that biological activities of various miRNAs contribute to invasion and metastasis in TSCC. Thus, determination of the functional and clinical importance of specific miRNAs may provide effective management of TSCC. Previous studies have demonstrated that miR-488 plays a tumor suppressive role in several cancers, including ovarian cancer [48], colorectal cancer [49], hepatocellular carcinoma [23], non-small-cell lung cancer [22] and gastric cancer [50].

In this study, for the first time we found that the level of miR-488 was significantly downregulated in TSCC tissues and cells. To test the biological function of miR-488 in TSCC, we overexpressed or knocked down miR-488 in TCA8113 cells by transfecting them with miR-488 mimics or inhibitors, respectively. Our transwell assay showed that the overexpression or knockdown of miR-488 dramatically suppressed or promoted the invasion of TCA8113 cells compared with the miR-NC group, respectively. Moreover, the expressions of MMP-2, MMP-7 and MMP-9 were significantly decreased, and the expressions of TIMP-1 and TIMP-2 were significantly increased in TSSC cells after transfection with a miR-488 mimic. Next, we assessed the changes in the EMT markers in TCA8113 cells transfected with a miR-488 mimic and inhibitor. Our data demonstrate that the upregulation of miR-488 could significantly increase the level of the epithelial marker E-cadherin and decrease the mesenchymal markers N-cadherin and vimentin. This suggests that miR-488 might reverse the EMT process to suppress cell invasion and metastasis.

No previous studies demonstrated a relationship between miR-488 and ATF3 in TSCC. Our findings show that the overexpression of miR-488 reduced the expression of ATF3 and inhibited cancerous signals such as invasion and EMT. Furthermore, restoration of ATF3 reversed the inhibitory effects of miR-488, indicating that miR-488 inhibited the invasion and EMT of TSCC cells through regulation of ATF3, and that ATF3 might play critical roles in metastasis of TSCC.

## Conclusions

Our results show that the expression of ATF3 was significantly upregulated and miR-488 level was dramatically downregulated in TSCC tissues. Overexpression of miR-488 inhibited invasion and EMT of TSCC cells through direct downregulation of ATF3 expression. Therefore, our study provided functional evidence to fully support the hypothesis that miR-488 and ATF3 are prognostic factors for TSCC.

## Abbreviations

ATF3: Transcription factor 3
CREB: cAMP responsive element-binding
EMT: Epithelial–mesenchymal transition
miRNA: microRNA
MMP: Matrix metalloproteinase
TSCC: Tongue squamous cell carcinoma
